The article "Deep Learning-Based Emergency Care Process Reengineering of Interventional Data for Patients with Emergency Time-Series Events of Myocardial Infarction" was retracted in 2023. Reasons: signs of a paper mill; suspected computer-generated content; unreliable results or conclusions; lack of ethics approval or compliance.

# Deep Learning-Based Emergency Care Process Reengineering of Interventional Data for Patients with Emergency Time-Series Events of Myocardial Infarction

**DOI:** 10.1155/2022/7339930

**Published:** 2022-02-23

**Authors:** Na Gao, Yue Xu, Lili Tu, Siyue Zhu, Shuhong Zhang

**Affiliations:** ^1^Department of Cardiology, The Second Medical Center and National Clinical Research Center for Geriatric Diseases, Chinese PLA General Hospital, Beijing 100853, China; ^2^Health Department, The Second Medical Center and National Clinical Research Center for Geriatric Diseases, Chinese PLA General Hospital, Beijing 100853, China; ^3^Emergency Department, The Second Medical Center and National Clinical Research Center for Geriatric Diseases, Chinese PLA General Hospital, Beijing 100853, China

## Abstract

This paper proposes a representation learning framework HE-LSTM model for heterogeneous temporal events, which can automatically adapt to the multiscale sampling frequency of multisource heterogeneous data. The proposed model also demonstrates its superiority over other typical approaches on real data sets. A controlled study is performed according to computerized randomization, with 38 patients in each of the two groups. The study group has a higher resuscitation success rate and patient satisfaction than the conventional group (*P* < 0.05), and the time from the first consultation to the completion of the first ECG, the time from the completion of the ECG to the activation of the path lab, and the time from the emergency admission to the balloon dilation were significantly shorter in the study group than in the conventional group (*P* < 0.05). The emergency care process reengineering intervention helps patients with acute myocardial infarction to be treated quickly and effectively, thus improving their resuscitation success rate and satisfaction rate, and is worthy to be caused in the clinic and widely applied.

## 1. Introduction

Acute myocardial infarction is a serious type of coronary heart disease, mainly caused by the complete occlusion of coronary arteries resulting in the interruption of myocardial blood perfusion and acute myocardial ischemic and hypoxia necrosis, which is sudden in onset, and as the area of myocardial infarction continues to expand, patients are prone to complications such as heart failure, arrhythmias, and other cardiovascular adverse events, which seriously threaten patients' lives [1]. As the condition of patients with acute myocardial infarction progresses rapidly and has a high risk of death, patients need to be treated promptly after the onset of the disease. Emergency intervention is a common treatment for acute myocardial infarction, which can effectively restore coronary perfusion, relieve myocardial ischemia, and achieve the purpose of controlling the condition.

In clinical practice, acute myocardial infarction is a relatively common condition caused by myocardial infarction due to insufficient oxygenation of the coronary arteries. It has a rapid onset and is very dangerous, manifesting as persistent and severe retrosternal pain, with a high mortality rate, and is easily complicated by shock, severe arrhythmia, and heart failure, having a serious impact on the physical and mental health of patients [2]. Opening the infected vessel as soon as possible is the key to successful clinical management of patients with acute myocardial infarction [3].

This paper presents a deep learning-based learning framework for the representation of patient electronic medical record data for the task of predicting clinical endpoints (clinical endpoints). Clinical endpoints are characteristics or target variables that reflect the patient's sensation, function, and survival. Research has demonstrated that deep learning has superior performance over traditional machine learning methods in various application scenarios, such as image classification [4], speech recognition [5], and natural language processing [6]. The main idea of deep learning is to automate the extraction of features from the underlying data to obtain an effective semantic representation of the sample. In the context of electronic medical records, it is also desirable to learn effective representations of patient history by means of deep learning. However, the patient history data representation learning problem is very challenging because patient history records contain heterogeneous temporal events, such as laboratory results, physiological indicators, drug injections, and clinical events. The frequency of sampling records varies widely from event to event; for example, patients may have their blood glucose tested every morning and their temperature and blood oxygen measured every hour [7]. There are also complex temporal dependencies between the different events; for example, a diagnosis can only be made based on some of the patient's previous symptoms and some trends in the laboratory results. As can be seen, learning vector representations of such heterogeneous temporal events, which contain thousands of events, vary greatly in sampling frequency, and imply a wealth of temporal dependencies, is indeed very complex [8].  Figure 1 shows representation learning modelling framework for heterogeneous temporal events.

However, during acute myocardial infarction emergency interventions, patients are affected by their condition, their psychological condition is not optimistic, is prone to anxiety, depression, and other negative emotions, and has a risk of cardiovascular events after interventions, which is not conducive to patient prognosis and requires patient care measures to intervene [9]. In recent years, the clinical medical model has gradually changed to a bio-psycho-social medical model, and the influence of psychological factors in the treatment has become more and more obvious, and clinical attention to the psychological condition of patients has become increasingly important. Dual-hearted care is a new nursing model that integrates the concept of dual-hearted medicine and advocates targeted nursing interventions for patients with mental and psychological disorders in cardiovascular disease, and its nursing measures are highly targeted and fully reflect the concept of person-centered care [10].

Much of the literature explores representation learning methods for sequential data, particularly in the speech and natural language processing domain [11]. Existing classical long short-term memory (LSTM) models can be used for homogeneous sequence data; however, it is not convenient to use LSTM models directly for heterogeneous sequence data. There is also some work (e g., Gaussian model [12]) to model the correlation between different sequences; however, its computational complexity is very large and computationally unaffordable when dealing with thousands of temporal data. Therefore, the author would like to find a method that can both model different events, with different sampling frequencies, and capture the correlation between different events and can be relatively easily extended for application to high-dimensional medical case data [13].

In another algorithmic model called heterogeneous event long short-term memory, HE-LSTM network is proposed as an algorithmic model for learning the joint representation of heterogeneous temporal events. The algorithm in this paper is based on sparsely updated recurrent neural networks such as the phased LSTM [14]. The phased LSTM deals with irregular event sequence data, using a phase gate to integrate data collected by sensors with arbitrary sampling frequencies, but it cannot be used directly for heterogeneous time-series event data from electronic medical records containing thousands of event types. Modelling a large number of heterogeneous events with widely varying sampling frequencies, each event and its attributes are embedded in a vector representation that is then fed into the HE-LSTM model, which relies on a division of labor between event gates to asynchronously track the timing information of certain clusters of related events at different sampling frequencies, so that the final learned joint representation can be automatically integrated using a hidden layer delayed update model structure to capture the various types of heterogeneous events. The final learned joint representations can then be automatically integrated with the help of the hidden layer delayed update model structure, which captures the timing dependencies associated with each type of event [15].

In this study, the observation group was given double-hearted care, and psychological care measures such as psychological guidance, psychological balance reconstruction, emotion adjustment training, role model motivation, and affection support were implemented to address the mental and psychological barriers of patients with acute myocardial infarction during emergency intervention. Quality of life scores were higher in the observation group than in the control group, indicating that double-hearted care can not only reduce the adverse emotions of patients with acute myocardial infarction, but also reduce the risk of cardiovascular events and the interference of adverse emotions and conditions on their quality of life, mainly because the care measures in the double-hearted care program are relatively comprehensive, among which, psychological diversion is mainly aimed at the adverse emotions of patients, which can pacify patients' dysphoria to make them as calm as possible.

The idea of this paper is not to make the initial division based on data in the form of cases, but to model events in the medical process as the basic unit, retaining the precise time of occurrence of the events. This allows for greater retention and reflection of the relationships between individual events and the frequency structure of different event occurrences. In this paper, when comprehensively modelling electronic medical record data using a representation learning framework for heterogeneous temporal events, all case information is treated as clinical events with attributes and ordered by time, while retaining the precise time of occurrence of events. While this allows for the full fusion of heterogeneous temporal events, the sequences consisting of heterogeneous events are very long, with the vast majority of patient samples in the MIMIC-III dataset having sequences over 10,000 in length. The difficulty of extracting complex temporal dependencies of heterogeneous temporal events then translates into the problem of maintaining long-term dependencies of ultra-long sequences.

## 2. Related Work

Another large body of work deals with case data by ignoring information about attributes in clinical events and using only discrete variables of clinical events (e.g., sequences of ICD codes) to predict clinical endpoints [16]. For example, some work trains separate semantic embedding vectors for different types of clinical events and then integrates them to predict subsequent drug abuse events (ADEs) [17]. Chang et al. [18] used two recurrent neural networks to generate attention weight for each ICD code during each patient visit, weighting the embedding vectors for the original ICD codes and then predicting the probability of occurrence of heart failure. There is also work using convolutional neural networks to model irregular sequences of medical codes to predict the risk of future morbidity [19]. Patient representation learning using deep learning techniques mainly follows the traditional event sequence and multivariate time series modelling approaches to independently model various types of data in cases. For example, the Google team proposed a fast healthcare interoperability resources (FHIR) storage format for such unprocessed data and used this format as the basis for deep learning modelling to predict a variety of important outcome events [12]. At the level of the basic format of electronic medical records, the approach in this paper coincides with it, not only in that it can be loosely adapted to the case record format of individual hospitals and solve the prediction problem, but also in that it does not lose important information due to data regularization.

To facilitate modelling, traditional work on clinical endpoint prediction has generally used only part of the electronic medical record data, thus avoiding direct treatment of heterogeneous time-series events. Some work has used, with expert guidance, only a subset of all medical events as patient characteristics [20]. For example, Sehatzadeh et al. [21] used 21 time series physiological signals (including 11 physiological indicators as well as 10 laboratory results) to predict intensive care unit (ICU) referrals. They had also selected 50 time series and modelled this subset of electronic medical record information with a multitasking Gaussian process, using the hypermastigote of the multitasking Gaussian process as a vector of representations of patients, in which predictions are made either by calculating patient similarity or by feeding into a conventional classifier in this vector space. It is worth noting that manual selection of some of the features introduces a passive export bias (export bias) and only reflects part of the information in the electronic medical record data. This type of work is difficult to fully exploit the information in the EHR as a whole [22].

However, of the EHR modelling level, traditional approaches model discrete data (e.g., ICD diagnosis codes) and continuous time series variables (e.g., blood pressure time series) separately, depending on the type of data. For example, the feed forward model with time-aware attention directly models the representation vector of a discrete event sequence, while the boosted embedded time series model models the representation vector of each time series. Model for each time series enumerates ten types of temporal predicates (e.g., values greater than V after a certain point in time *T*, etc.), and finally 100,000 predicates are filtered and fed into the neural network as features. In the processing of recording time, intervals are usually used to give a uniform timestamp to events with fixed time intervals; for example, the weighted recurrent neural network [23] (weighted RNN) model divides discrete event series data into 10 broad categories, fixes 12 h as the time interval, divides the series into sequences of event groups, learns vector representations for each category of sequences separately, and integrates them at the level of prediction results output.

## 3. Model Design

### 3.1. Problem Definition

Given a patient *p* in the electronic patient record data, the features of *p* are composed of dynamic features of sequence length N {*X*_*t*_}_1≤*t*≤*N*_. {*X*_*t*_}_1≤*t*≤*N*_ can be viewed as a heterogeneous sequence of medical events, *X*_*t*_ as a triple *X*_*t*_ = (type, value, time), type being the type of event, value being the attribute of the event, and time being the time at which the event was recorded. The events in {*X*_*t*_}_1≤*t*≤*N*_ are arranged in chronological order. The event type vector is denoted as *e*=*X*_*t*_.*type*. Patient *p* corresponds to a binary label 0 or 1, indicating a clinical endpoint event that occurred at *X*_*N*_ time +24h, such as a stable condition or patient death.

The goal of this paper is to dynamically predict two important clinical outcomes based on historical clinical data (heterogeneous time-series events) of patients. The first task is death prediction, which predicts whether a patient is still receiving treatment or has died. The second task is the prediction of abnormal potassium concentrations, the goal of which is to confirm whether the blood potassium assay is an abnormal value.

### 3.2. Event Embedding

For event *X*_*t*_=(type, value,  time)  at time *t*, encode type and value separately. Type vector is a one-hot vector. Let *C*_type_ ∈ *R*^*N*×*M*^ be the encoding matrix of type, where N is the number of dimensions after encoding and *M* is the number of type categories; then, the encoding of type is

(1) $$\begin{array}{c} p=C_{\text{type}}\times \text{type}. \end{array}$$

The event attribute value consists of two parts: value = [value C, value n]. Both are also unique heat vectors, with value C being the discrete variable attribute of the event and value *n* being the numerical attribute. Again, denote their encoding matrices by *V*_*C*_ ∈ *R*^*N*×*C*^, *V*_*N*_ ∈ *R*^*N*×*U*^, respectively, where U is the total number of discrete attributes and C is the total number of continuous attributes. The encoding of the attributes is summed with the event type *p* to obtain the overall encoding of the dynamic event:

(2) $$\begin{array}{c} x_{d}=p+V_{c}\times {\text{value}}_{c}+\tanh\left(V_{n}\times {\text{value}}_{n}\right). \end{array}$$

*V*_*c*_, *V*_*n*_, and *C*_*type*_ are the parameters to be learned.

### 3.3. Heterogeneous Event LSTM

Figure 2 shows the basic structure of the neuron in HE-LSTM. The main difference between the two is that there are three gate functions in the base LSTM neuron, namely, input gate, output gate, and forget gate.

The core idea of the HE-LTSM model is to divide and conquer. The neurons track the information of different event clusters in different cycles and asynchronously. Based on the classical LSTM, an event gate *j*_*l*_ (the subscript *l* indicates the first input and *j*_*l*_ takes the value 0 or 1) is designed for each hidden layer neuron, which is updated normally according to the LSTM if it is turned on, and remains unchanged if it is turned off, as shown in (3), where the update value is calculated by the classical LSTM.

(3) $$\begin{array}{c} c_{l}=j_{l}{\tilde{c}}_{l}+\left(1-j_{l}\right)c_{l-1},\\ {\tilde{c}}_{l}=f_{l}c_{l-1}+i_{l}\tanh\left(W_{cx}x_{l}+W_{ch}h_{l-1}+b_{c}\right). \end{array}$$

The event gate *j*_*s*,*t*_ determines the switching state by the event type S and the time *t* at which the event is recorded. Equation (4) is an expression for event gate *j*_*s*,*t*_. It consists of two parts, an event filter (determined by event type S) and a phased gate *k*_*t*_ (determined by time t):

(4) $$\begin{array}{c} j_{s,t}=e_{s}k_{t}. \end{array}$$

The event filter allows only certain types of events to be fed into the neuron, and the phase gate allows the neuron to be open only for certain periods. This ensures that each neuron will only capture and sample the features of certain types of events, solving the problem of complex temporal diversity and poor training results caused by long sequences of medical events. The expression for the event filter is shown in (5).

*σ*(-) denotes the sigmoid function, tanh(-) denotes the hyperbolic tangent function, *W*_*ms*_, *W*_*em*_ are the matrix parameters learned in training, and *b*_*m*_, *b*_*e*_ are the vector parameters learned in training. Event filters allow each neuron to focus on a different set of events and thus better to learn the information in the mixed event sequence.

(5) $$\begin{array}{c} e_{s}=\sigma \left(W_{em}\tanh\left(W_{ms}s+b_{m}\right)+b_{e}\right). \end{array}$$

The phase gate *k* is a periodically varying function, as shown in (6). Given an initial phase *s* of period *τ*, *k*_*t*_ is a function of *ϕ*_*t*_, which also varies with *t* with a period of *τ*. Run is a hypernatremia that controls the proportion of the full period that the open state of the phase gate accounts for. At 0 < *ϕ*_*t*_ < *r*_on_, the phase gate is open; at other moments, since it is again a hypernatremia very close to 0, *k*_*t*_ is close to 0 and the phase gate is closed. All parameters can be updated only when the phase gate is open, so that the input can be sampled periodically, thus solving the problem of overly long input sequences.

(6) $$\begin{array}{c} \phi_{t}=\frac{\left(t-s\right)\mathrm{mod}\tau }{\tau },\\ k_{t}=\left\{\begin{array}{c} \frac{2\phi_{i}}{r_{\text{on}}},\phi_{i}<\frac{1}{2}r_{\text{on}},\\ 2-\frac{2\phi_{t}}{r_{\text{on}}},\frac{1}{2}r_{\text{on}}<\phi_{t}<r_{\text{on}},\\ \alpha \phi_{t}. \end{array}\right) \end{array}$$

In summary, for a certain neuron, the information about the events in its sampling cycle will only be updated into the neuron if it meets the type conditions of the corresponding event gate, so it can be considered that this neuron represents the state of a certain class of events at a certain sampling cycle.

Equation (7) is the loss function, which takes the form of cross-entropy. *y*_*t*_ is the prediction result of the model at moment *t*, ${\hat{y}}_{t}$ denotes the true indicator, and N is the total number of training samples. In (8), *h*_*t*_ is the output of the hidden layer at moment *t*, and *w*_*p*_ and *p*_*b*_ are the vector parameters to be learned in training.

(7) $$\begin{array}{c} \mathrm{Loss}\left({\hat{y}}_{t},y_{t}\right)=\frac{1}{N}\sum_{1\leq i\leq N}\left({\hat{y}}_{t}\times \;\ln\;y_{t}+\left(1-{\hat{y}}_{t}\right)\times \;\ln\left(1-y_{t}\right)\right). \end{array}$$

(8) $$\begin{array}{c} y_{t}=\mathrm{sigmoid}\left(w_{p}h_{t}+p_{b}\right). \end{array}$$

## 4. Case Studies

### 4.1. General Information

A total of 76 patients with acute myocardial infarction who received emergency intervention in a tertiary hospital from December 2018 to December 2019 were selected as the research objects. A controlled study was conducted according to computerized randomization, with 38 patients in each of two groups, one of which was called the conventional group and the other the study group. The study group consisted of 20 males and 18 females, aged 43–85 years, mean (63.2 ± 5.8) years, with an onset-to-admission time of 1–2 h, mean (1.4 ± 0.6) *h*. The conventional group consisted of 21 males and 17 females, aged 42–86 years, mean (63.6 ± 5.9) years, with an onset-to-admission time of 0.5–2 h, mean (1.5 ± 0.7) *h*. The basic data of each group were tested by clinical statistics, and the results had a *P* value > 0.05, which is of high value for the study.

Figure 3 shows the emergency care process reengineering diagram. (1) The success rate of resuscitation is recanalization of the infected vessel, stenosis residual less than 50%, and blood flow to grade III; (2) patient satisfaction is evaluated on the Likert scale [8], with 5 being very satisfied, 4 being more satisfied, 3 being fair, 2 being dissatisfied, and 1 being extremely dissatisfied; total satisfaction = very satisfied + relatively satisfied + fair; (3) time from first consultation to completion of the first ECG, time from completion of ECG to activation of the catheterization laboratory, time from emergency admission to balloon dilation were recorded for patients in the study group and the conventional group.

### 4.2. Results

The study group successfully resuscitated 35 cases (92.11%), and the conventional group successfully resuscitated 30 cases (78.95%). The difference between the groups was significant (X2 = 14.107, p  <  0.05).  Table 1 shows comparison of satisfaction between the study group and the conventional group.

The study group had a higher satisfaction rate of 94.74%, which was significantly different from the conventional group (*p* < 0.05).  Table 2 is comparison of emergency time (min) between the study group and the conventional group.

## 5. Experimental Results

### 5.1. Data Description and Experimental Setup

The experiments in this paper were conducted on a death prediction dataset and an abnormal lab result prediction potassium ion abnormality prediction dataset generated from ICU patient chart data (MIMIC-III [24]) from a US medical health centre (Beth Israel Deaconess Medical Center). The dataset was drawn from a sample of 24,301 patients from MIMIC-III, covering a total of 3,418 species with a total of 20,290,879 heterogeneous time-series events, with an average time span of 87 h 58 min.

### 5.2. Comparison Methods

In this paper, HE-LSTM is compared with three types of approaches: independent sequence models (independent LSTM, independent LSTM with shared parameters), delayed update recurrent neural network models (e.g., clock-work RNN, phased LSTM), and heterogeneous sequence models in the medical field (LSTM + event embedding, Retain). The clock-work RNN and phased LSTM were introduced in the previous section.

### 5.3. Evaluation Indicators

Since the dataset has the problem of positive and negative sample imbalance, this paper uses AUC (the area under ROC curve) and AP (average precision [25,26]) as evaluation indicators. Both are tenacious and robust for data with positive and negative sample imbalance.

### 5.4. Quantifying Experimental Results

Table 3 demonstrates the respective AUCs and APs of the different methods on the mortality prediction and abnormal laboratory results prediction datasets. The following conclusions can be drawn from the data in Table 3. Firstly, it is possible to model the correlation between the different event models. Overall, they were better than those modelling temporal data sampled from each data source individually, with HE-LSTM achieving the best performance results. For example, in the patient mortality prediction task, Retain, LSTM + event embedding, and HE-LSTM yielded improvements in AP of 0.0235, 0.1872, and 0.2114, respectively, relative to the best performing independent sequential model (independent LSTM). Consistent results were also found for other datasets and rubrics. And the models in this paper achieved the best results on such heterogeneous event sequence models. For example, HE-LSTM improved the AP on abnormal laboratory outcome prediction by 0.0818 and 0.0893 compared to Retain and LSTM + event embedding. It can be concluded that the correlation dependencies of heterogeneous time series of events are very effective for clinical endpoint prediction; learning the joint distribution of different events can effectively capture the time series of different events compared to the events independently [27].

Secondly, models that can adapt to newer sampling frequency coefficients are superior compared to densely updated RNNs. For example, the clock-work RNN improves AP in 0.1608 and 0.188, respectively, on the death prediction experiment compared to the independently modelled sequence model. Also, the phased LSTM improves AUC by 0.0526 and AP in 0.0606 on the abnormal lab prediction outcome task relative to the best performing independent sequence model (independent LSTM). It is possible to conclude that models with multiple frequency sampling are also useful for predicting clinical endpoints and that sparsely updated models can take advantage of this property by allowing different units to focus on more important inputs, rather than treating all inputs in a long sequence equally.

Moreover, the HE-LSTM achieves the highest performance on different datasets and different evaluation metrics. The HE-LSTM outperforms not only the sparse update RNN model but also the heterogeneous sequence model. Neither sparse update models, which only exploit the multifrequency sampling feature, nor heterogeneous sequence models, which directly conflate all different types of events, are the best choice for clinical endpoint prediction. For example, HE-LSTM improves the AUC by 0.1116 and the AP by 0.0506 on the death prediction task compared to the best sparse update model (clock-work RNN). Meanwhile, on the abnormal laboratory result prediction task, HE-LSTM improves the AUC and AP by 0.0662 and 0.0818, respectively, compared to the heterogeneous event sequence model Retain. It can be concluded that HE-LSTM achieves the best prediction performance due to tracking the temporal dependence of different events and automatically adapting to different sampling frequencies for different events as follows.

### 5.5. Comparison of Model Effects for Different Input Sequence Lengths

In order to verify the ability of the model proposed in this paper, as well as other sequence models, to capture the temporal dependence of heterogeneous events, the model is fed with sequence data of different lengths ranging from 20 to 1000 events. The following conclusions can be drawn from Figure 4. First, temporal sequence information is effective in predicting clinical endpoints. Most models improve in effectiveness as the length of the input sequence increases, especially when the input length is less than 200.

Second, HE-LSTM is better at capturing temporal dependencies in heterogeneous temporal events than other models. When the input length is small, each model behaves similarly, in which case the temporal dependencies are essentially cooccurring relationships of events occurring over the same period of time. Thus, the combination of individual event representation vectors and the joint representation of heterogeneous events responds with essentially the same amount of information. However, the performance of the model steadily improves as the sequence length exceeds 200 and gets longer (AP from 0.755 to 0.769 and AUC of 0.948 to 0.952). In contrast, the other models largely did not improve particularly well because they could not capture the temporal dependencies under very long sequences relatively well. Figure 4 is schematic comparison of model effects for different input sequence lengths.

### 5.6. Comparison of the Effects of Different Initialization Cycles

In order to explore the role of event filters in event gating, this paper compares the role of HE-LSTM with that of a model with event filters removed (i.e., phase gating only). The death prediction task was trained with different initialization periods given to the model, which were exponentiation with four uniform distributions: exp(U(1,2)), exp(U(2,3)), exp(U(3,4)), and exp(U(4,5)).

Figure 5 reflects the performance of the two models with different dimensions of the event embedding and the type of gates set in the model. For example, “32 phase gates” mean that the dimension of the event embedding vector is 32 and the model contains only phase gates; “64 event gates” mean that the event embedding dimension is 64, which is the full HE-LSTM model. The full HE-LSTM is tenaciously robust to different initialization cycles. For example, with the four initialization settings mentioned above, the full HE-LSTM improves the AP on the death prediction task by 0.025, 0.028, 0.018, and 0.042 on average compared to the model without event filters. It can therefore be concluded that event dates can be more easily adapted to multiscale sampling frequencies of heterogeneous temporal events due to the help of event filters. Figure 5 reflects comparison of the effects of different initialization cycles.

Acute myocardial infarction is relatively common in clinical practice. The disease is fast developing and has a high risk of death, and an efficient, fast, and reasonable scientific emergency care process is an important guarantee for clinical life savings of patients' safety [25]. However, under the conventional care model, the procedures are cumbersome and many norms are unreasonable, which can easily delay the best time for patients to be rescued and treated [26]. The emergency department of our hospital intervened in patients with acute myocardial infarction by reengineering the emergency care process, reducing the complicated process into a simple one, and shortening the time spent on registration and payment and waiting for medical orders [27]. The reengineering of the emergency care process was compiled in a booklet, making it easier for nursing staff to follow the protocols, avoiding oversights or omissions due to differences in work capacity and responsibility, and ensuring the effective implementation of all emergency strategies [28]. In the process of emergency interventions, nursing staff are required to actively participate in the process, to feel that “time is life”, to enhance their sense of mission and responsibility, and to increase their motivation and initiative in the process of reengineering the emergency care process [29, 30]. At the same time, nursing staff were required to actively participate in the postoperative observation and follow-up work to understand the feelings of patients and their families about the new nursing process, to actively communicate with patients under the new process model, and to actively listen to their opinions or suggestions, to reduce patients' negative psychology and eliminate their worries and concerns [31]. Therefore, the satisfaction rate of the study group was higher than that of the conventional group (*P* < 0.05). It is suggested that emergency care process reengineering can significantly improve the satisfaction of patients with acute myocardial infarction [32].

In conclusion, for patients with acute myocardial infarction treated by emergency intervention, the reengineering of the emergency care process can further improve their resuscitation success rate and satisfaction rate and shorten their emergency waiting time, which is worthy of great reference in clinical practice [33].

## 6. Conclusions

In this paper, we propose a representation learning framework HE-LSTM model for heterogeneous temporal events, which can automatically adapt to the multiscale sampling frequency of multisource heterogeneous data, and by tracking the temporal information of different events asynchronously, the patient representation vector obtained from this model can capture the temporal dependencies between different times. And the model in this paper also demonstrates its superiority over other typical approaches on real data sets.

Furthermore, the framework can be transferred to other domains, especially for applications such as sensor data or behavioral recording data sampled asynchronously from multiple sources. For example, the framework can be used to model representational learning of user behavior in recommending systems research or representational learning of student learning behavior in smart education research.

## Figures and Tables

**Figure 1:** Representation learning modelling framework for heterogeneous temporal events.

**Figure 2:** Basic structure of neurons in HE-LSTM.

**Figure 3:** Flow chart for reengineering emergency care.

**Figure 4:** Schematic comparison of model effects for different input sequence lengths. (a) AUC of different models. (b) AP of different models.

**Figure 5:** Comparison of the effects of different initialization cycles. (a) AUC of different models. (b) AP of different models.

**Table 1:** Comparison of satisfaction between the study group and the conventional group.

Group	Number of cases	Very satisfied	Quite satisfied	General satisfaction	Dissatisfied	Extremely dissatisfied	Total satisfaction
Research group	38	18 (47.37%)	10 (26.32%)	8 (21.05%)	2 (5.26%)	0	36 (94.74%)
General group	38	12 (31.58%)	9 (23.68%)	9 (23.68%)	5 (13.16%)	3 (7.89%)	30 (78.95%)
*χ* ^2^	-						15.192
P	-						<0.05

**Table 2:** Comparison of emergency time (min) between the study group and the conventional group.

Group	Number of cases	Completion time from the first diagnosis to the first ECG	Time from completion of ECG to activation of catheter room	Time from emergency admission to balloon dilatation
Research group	38	5.3±1.6	22.1±2.8	66.5±10.4
General group	38	10.4±1.7	45.6±4.9	93.5±9.8
t	-	26.550	42.158	22.391
p	-	<0.05	<0.05	<0.05

**Table 3:** Experimental results for prediction of death and prediction of abnormal laboratory results.

Method	Death prediction		Potassium ion anomaly prediction	
	AUC	AP	AUC	AP
Independent LSTM	0.8771	0.5573	0.7196	0.2969
Independent LSTM with shared parameters	0.8064	0.5301	0.5308	0.1098
Phased LSTM	0.8474	0.4900	0.7722	0.3575
Clock-work RNN	0.8400	0.7181	0.6516	0.2208
Retain	0.8967	0.5808	0.7325	0.3096
LSTM + event embedding	0.9466	0.7445	0.7231	0.3021
HE-LSTM	0.9516	0.7687	0.7987	0.3914

## Data Availability

The simulation experiment data used to support the findings of this study are available from the corresponding author upon request.
